# Specific Inhibition of Tumor Cells by Oncogenic *EGFR* Specific Silencing by RNA interference

**DOI:** 10.1371/journal.pone.0073214

**Published:** 2013-08-08

**Authors:** Masaki Takahashi, Tomoko Chiyo, Takashi Okada, Hirohiko Hohjoh

**Affiliations:** 1 Department of Molecular Pharmacology, National Institute of Neuroscience, National Center of Neurology and Psychiatry, Kodaira, Tokyo, Japan; 2 Department of Molecular Therapy, National Institute of Neuroscience, National Center of Neurology and Psychiatry, Kodaira, Tokyo, Japan; Institute of Medical Science, University of Tokyo, Japan

## Abstract

Anticancer agents that have minimal effects on normal cells and tissues are ideal cancer drugs. Here, we show specific inhibition of human cancer cells carrying oncogenic mutations in the epidermal growth factor receptor (EGFR) gene by means of oncogenic allele-specific RNA interference (RNAi), both *in vivo* and *in vitro*. The allele-specific RNAi (ASP-RNAi) treatment did not affect normal cells or tissues that had no target oncogenic allele, whereas the suppression of a normal *EGFR* allele by a conventional *in vivo* RNAi caused adverse effects, i.e., normal EGFR is vital. Taken together, our current findings suggest that specific inhibition of oncogenic *EGFR* alleles without affecting the normal *EGFR* allele may provide a safe treatment approach for cancer patients and that ASP-RNAi treatment may be capable of becoming a safe and effective, anticancer treatment method.

## Introduction

The *EGFR* gene has various nucleotide variations, some of which are oncogenic; and oncogenic *EGFR* nucleotide variants have been identified as causative agents in a variety of cancer types [1]. For example, lung cancer, which is the most common cancer and affects an increasing number of cancer patients [2], appears to be closely related to mutant EGFR. Approximately 80% of lung cancer cases are classified as non-small-cell lung cancer (NSCLC), and many NSCLC cases involve an *EGFR* mutation [1,3]. A common oncogenic *EFGR* mutation is the deletions of exon 19, which appear to promote EGFR tyrosine kinase activity [4,5]; and such deletion mutants account for 45%, or more, of NSCLC cases in Asia [1,3].

Specific inhibition of oncogenic *EGFR* alleles may be a promising strategy for therapy for cancer patients carrying causative oncogenic *EGFR* mutations. Gefitinib and erlotinib are well-known EGFR-tyrosine kinase inhibitors (EGFR-TKIs), and are each currently used as an anticancer drug in the treatment of cancers [6–8]. In addition to such EGFR-TKIs, another agent that has an inhibitory mechanism different from EGFR-TKIs against mutant EGFR, if any, may be useful and necessary for responding to various cancers; and such different agents may compensate for their imperfection to each other in anticancer therapies.

Allele-specific RNAi (ASP-RNAi) is an atypical RNAi silencing that is capable of discriminating between target (mutant) and non-target (wild-type) alleles, and may be an applicable tool in specific inhibition of disease-causing alleles, i.e., disease-causing allele-specific RNAi. The disease-causing allele-specific RNAi may provide us with a novel treatment strategy different from treatments with EGFR-TKIs.

For induction of ASP-RNAi, the design and selection of small interfering RNAs (siRNAs) that confer ASP-RNAi are vital, but quite difficult. However, our *in vitro* assay system for assessment of siRNAs substantially mitigated the difficulty [9–13].

In this study, we focused on *EGFR* deletions to discriminate between oncogenic *EGFR* alleles and the normal *EGFR* allele, and designed siRNAs that targeted the oncogenic *EGFR* mutations for ASP-RNAi. Our findings indicated that ASP-RNAi-mediated silencing of disease-causing *EGFR* alleles specifically inhibited the proliferation of human cancer cells carrying the oncogenic alleles, but did not affect normal cells or tissues that had no target oncogenic allele *in vivo*.

## Materials and Methods

### Cell culture

The PC-3 and PC-9 human non-small-cell lung cancer cell lines were obtained from Health Research Resources Bank (JCRB No.JCRB0077) and Immuno-Biological Laboratories (No. 37012), respectively. Both cell lines were grown in RPMI-1640 medium (Invitrogen, Carlsbad, CA, USA) supplemented with 10% fetal bovine serum (Invitrogen), 100 units/ml penicillin, and 100 µg/ml streptomycin (Wako, Osaka, Japan) at 37° C in a 5% CO_2_ humidified chamber. HeLa cells were grown in Dulbecco’s modified Eagle’s medium (DMEM) (Wako) supplemented with 10% fetal bovine serum (Invitrogen), 100 units/ml penicillin, and 100 µg/ml streptomycin (Wako) at 37° C in a 5% CO_2_ humidified chamber.

### Mice

BALB/c nu/nu male mice (5-6 weeks old) and ICR male mice were purchased from CLEA Japan, Inc (Tokyo, Japan). Mice were housed, fed and maintained in the laboratory animal facility according to the National Institute of Neuroscience animal care guidelines. This study was carried out in strict accordance with the recommendations in the Guide for the Care and Use of Laboratory Animals of the National Institutes of Neuroscience. The protocol was approved by the Committee on the Ethics of Animal Experiments of the National Institutes of Neuroscience (Permit Number: 2012003).

### RNA and DNA oligonucleotides

DNA oligonucleotides and siRNAs used in this study were synthesized by and purchased from Sigma-Aldrich (St Louis, MO, USA).

### Purchased siRNAs

*Silencer*® Select Validated siRNAs targeting the normal mouse *Egfr* gene were purchased from Applied Biosystems (Carlsbad, CA, USA). The manufacturer’s IDs are s65373 and s65374, and the siRNAs were named siEgfr#01 (s65373) and siEgfr#02 (s65374). The siEgfr#01 siRNA was ultimately designated “siEgfr” in this study. A *Silencer*® Select Validated siRNA targeting the normal human *EGFR* gene was also purchased from Applied Biosystems. The manufacturer’s ID is s563, and the siRNA was named siEGFR.

### Transfection and reporter assay

Construction of reporter alleles, transfections, and the reporter assay were carried out as described previously [9–13]. The DNA oligonucleotide sequences of the mutant and wild-type (normal) *EGFR* alleles used in the construction of the reporter alleles, and the sequences of siRNAs are indicated in Tables S2 and S1, respectively. Briefly, the day before transfection, HeLa cells were treated with trypsin, suspended in fresh medium without antibiotics, and seeded onto 96-well culture plates at a cell density of 1 × 10^5^ cells/cm^2^. The pGL3-TK-backbone plasmid (60 ng), phRL-TK-backbone plasmid (10 ng), pSV-β-Galactosidase control vector (20 ng) (Promega, Fitchburg, WI, USA), and 20 nM (final concentration) of each siRNA duplex were added to each well; Lipofectamine2000 transfection reagent (Invitrogen) was used according to the manufacturer’s instructions. Cell lysates were prepared 24 h after transfection, and the expression levels of luciferase and β-galactosidase were examined using a Dual-Luciferase Reporter Assay System (Promega) and a Beta-Glo Assay System (Promega), respectively. The luminescent signals were measured using a Fusion Universal Microplate Analyzer (PerkinElmer, Waltham, MA, USA).

For the examination of dose-dependent inhibition of siRNA [50% inhibitory concentration (IC50) of siRNA], the pGL3-TK-backbone plasmid (60 ng), phRL-TK-backbone plasmid (10 ng), and pSV-β-Galactosidase control plasmid (20 ng) were added, along with various amount of each siRNA [0, 0.001, 0.005, 0.02, 0.08, 0.32, 1.25, 5, 10, and 20 nM (final concentration)], into each well; co-transfections were performed using Lipofectamine2000 transfection reagent (Invitrogen). The expression levels of luciferase and β-galactosidase were examined 24 h after transfection as described above. The data were fitted to the Hill equation (Hill coefficient; *n* = 1) and IC_50_ values were determined.

### Total RNA preparation and cDNA synthesis

Total RNAs were extracted from cultured human cells using TRIzol Reagent (Invitrogen). RNA samples were templates for cDNA synthesis, which was performed with Oligo(dT)_15_ primers (Promega) and a SuperScript III reverse transcriptase (Invitrogen) according to the manufacturer’s instructions.

### PCR analyses

PCR analysis was carried out using the primer sets described below and an AmpliTaq Gold DNA polymerase (Applied Biosystems, Carlsbad, CA, USA), according to the manufacturer’s instructions. The GeneAmp PCR system 9700 (Applied Biosystems) was used as a thermal cycler, and the thermal cycling profiles were as follows: heat denaturation at 95° C for 10 min, 30 cycles of amplification including denaturation at 98° C for 30 s, annealing at 55° C for 30 s, and extension at 72° C for 30 s. The resultant PCR products were separated by electrophoresis on 5% polyacrylamide gels and visualized by ethidium bromide staining.

The sequences of the PCR primers used were as follows.

EGFR deletion detection primer set:

5’ -CCCAGAAGGTGAGAAAGTTGAAATT-3’

5’ -TCATCGAGGATTTCCTTGTTGGC-3’

### Hoechst 33342 and propidium iodide (PI) staining

Hoechst 33342 (2 µg/ml, Cell signaling Technology, Danvers, MA, USA) and propidium iodide (2 µg/ml, Invitrogen) were added to the cultures to count total cells and dead cells, respectively. After incubation for 30 min at 37° C, the stained cells were examined using a ZEISS fluorescent microscope (Axiovert 40 CFL).

### Xenograft model and antitumor effects of intratumoral siRNA administration

PC-3 cells were treated with trypsin and resuspended in phosphate-buffered saline (PBS) containing 50% matrigel (BD Biosciences, San Jose, CA, USA) at a final concentration of 1 × 10^7^ cells/ml; 200 µl of cell suspension (≈2 × 10^6^ cells) were injected subcutaneously into the left flank of individual BALB/c nu/nu (nude) mice anesthetized by intraperitoneal injection of Somnopentyl (50 mg/kg b.w.). Tumor growth was measured with a caliper (details below). When tumors reached 100 mm^3^ or more in size, a one-time intratumoral siRNA administration was performed; siRNA was mixed with atelocollagen (AteloGene Local Use; Koken, Tokyo, Japan) according to the manufacturer’s instructions, and the resultant siRNA/atelocollagen complexes were administered (1.0 mg/kg b.w.: 20 µg siRNA /200 µl /injection). Treated tumors were measured with a caliper weekly for more than 4 weeks following siRNA administration. For each measurement, the longest and widest dimensions of the tumors were measured, and tumor volume was calculated using a conventional formula:

Tumor volume (mm^3^) = (length) × (width)^2^ × 0.5

To further monitor xenograft tumors *in vivo*, the *firefly luciferase* gene was introduced into PC-3 cells via a viral vector [14–16]. The resultant PC-3/luc cells were injected subcutaneously into athymic nude mice as in PC-3 cells. Xenograft tumors were treated with siRNAs at a dose of 0.5, 1.0 or 2.0 mg/kg b.w. and monitored by an IVIS imaging system (Xenogen, Alameda, CA, USA) according to the manufacturer’s instructions.

### Lung cancer model and antitumor assay by systemic siRNA administration

PC-3/luc cells (≈2 × 10^6^ cells/100 µl in PBS) were administered once a day for 3 days to athymic nude mice (male, 7-week-old) via the lateral tail vein. Three days (Day 3) after the final administration (Day 0), the mice were examined using an IVIS imaging system (Xenogen, Alameda, CA, USA) according to the manufacturer’s instructions; mice with luc-positive PC-3 cells were identified and randomly divided into two groups (6 mice/group). For systemic siRNA administration, the test and control siRNAs were each prepared with atelocollagen (AteloGene Systemic Use; Koken) according to the manufacturer’s instructions; the resultant siRNA/atelocollagen complexes (1.0 mg/kg b.w.) were administered twice (Day 5 and 7) to PC-3/luc-positive mice via the lateral tail vein. The experiments of siRNA administration with atelocollagen were designed by reference to the previous reports [17–20]. The treated mice were examined again using an IVIS imaging system: photographic images of the luminescent signal intensities were taken 10 min after injection of D-Luciferin (75 mg/kg b.w.) and the images were analyzed using a Living Imaging software (Xenogen).

To visualize apoptotic cells *in vivo*, VivoGlo Caspase 3/7 substrate (2 mg/200 µl) (Promega) was administrated intraperitoneally to the treated PC-3/luc-positive mice 6 h after the first injection of siRNAs, which occurred on Day 5; *in vivo* imaging and subsequent imaging analysis was carried out as described above.

### RNAi knockdown of the normal Egfr gene in vivo

*Silencer*® Select Validated siRNAs targeting normal mouse *Egfr* gene (Applied Biosystems, Carlsbad, CA, USA) (see Purchased siRNAs) were used. The siRNAs (siEgfr) were prepared with atelocollagen (AteloGene Systemic Use; Koken) as described above, and the siRNA/atelocollagen complexes (1.0 mg/kg b.w.) were administered 3 times, on Days 1, 3, and 5, to 10-week-old ICR mice (male) via the lateral tail vein. Two days after the last administration, the treated mice were sacrificed and subjected to toxicological, biochemical, and histological analyses.

### Western blot analysis

Cultured cells and tumors treated with indicated siRNAs were harvested and lysed in lysis buffer [20 mM Tris-HCl (pH 7.5), 150 mM NaCl, 1 mM EGTA, 1% Triton X-100] containing a 1× protease inhibitor cocktail (Protease Inhibitor Cocktail Tablets; Roche Diagnostics, Basel, Switzerland); protein concentration in each cell lysate was measured using a Protein Quantification kit (DOJINDO, Mashiki-town, Kumamoto, Japan). Equal amounts of protein (≈10 µg) were mixed with 4× sample buffer (0.25 M Tris-HCl, 40% glycerol, 8% SDS, 0.04% bromophenol blue, 8% beta-mercaptoethanol), boiled for 5 min, and then separated by SDS-PAGE on 10% polyacrylamide gels. After electrophoresis, separated proteins were blotted via electrophoresis onto polyvinylidene fluoride membranes (Immobilon P; Millipore, Billerica, MA, USA). The membranes were incubated for 1 h in blocking solution [5% bovine serum albumin (Sigma-Aldrich) in TBS-T buffer (TBS containing 0.1% Tween-20)] and then with diluted primary antibodies (described below) at 4° C overnight; membranes were then washed in TBS-T buffer, and further incubated with 1/5000 diluted horseradish peroxidase-conjugated goat anti-mouse IgG (Sigma-Aldrich) or goat anti-rabbit IgG (Sigma-Aldrich) for 1 h at room temperature. Antigen–antibody complexes were visualized using Immobilon Western Chemiluminescent HRP Substrate (Millipore). The primary antibodies used in Western blotting and their dilution ratios in parentheses were as follows:

anti-epidermal growth factor receptor (EGFR) (1/1000), anti-phospho-EGFR (1/1000), anti-EGFR (E746-A750del Specific) (6B6) (1/1000), anti-Akt (1/1000), anti-phospho-Akt (1/1000), anti-Erk1/2 (1/2000), and anti-phospho-Erk1/2 (1/2000) antibodies; all of these antibodies were purchased from Cell Signaling Technology. The anti-Tubulin antibody (1/10000) was purchased from Sigma Aldrich.

### Histochemical and immunofluorescence staining

Dissected tissues were washed with phosphate-buffered saline (PBS), fixed with 4% paraformaldehyde at 4° C for over 4 h, incubated in 20% sucrose/PBS at 4° C overnight, embedded in the O.C.T. compound (Sakura Finetech Japan, Koto-ku, Tokyo, Japan) on a dry ice/ethanol bath, and then cut into 15-µm-thick sections. Cryosections were fixed with cold methanol, permeated by 0.1% Triton-X100 in PBS, and incubated in blocking solution (4% BSA in PBS) for over 1 h. The pretreated cryosections were incubated with diluted primary antibodies (described below) at 4° C overnight, washed with PBS, and further incubated with 1/1000 diluted anti-rabbit IgG Alexa 555-conjugated antibody (Molecular Probes, Carlsbad, CA, USA) or anti-mouse IgG Alexa 488-conjugated antibody (Molecular Probes) at room temperature for 2 h. In addition, nuclear staining with Hoechst 33342 (Cell Signaling Technology) or PI (Invitrogen) was carried out. After washing with PBS, the cryosections were mounted in Fluorescent Mounting Medium (DakoCytomation, Glostrup, Denmark) and examined using a ZEISS fluorescent microscope (Axiovert 40 CFL). The primary antibodies and the associated dilution ratios and manufacturers in parenthesis were as follows:

anti-Ki67 antibody (1/500; EPITOMICS, Burlingame, CA, USA) and anti-CD31 antibody (1/500; BD Biosciences, San Jose, CA, USA).

For examination of apoptotic cells, a TdT-mediated dUTP Nick-End Labeling (TUNEL) assay was performed using the DeadEnd™ Fluorometric TUNEL System (Promega), according to the manufacturer’s instructions. A conventional H&E staining was also performed.

### Blood examination

Blood specimens were drawn from the lateral tail vein or abdominal aorta of mice. Red and white blood cells were counted using a hemocytometer. Hematocrit was measured in capillary tubes. Plasma specimens were subjected to biochemical analyses using the following commercial kits: assay kits for alkaline phosphatase (ALP), total protein (TP), GPT, and GOT were obtained from KAINOS laboratories inc. (Tokyo, Japan), and an assay kit for bilirubin (total, direct, and indirect) was obtained from BioAssay Systems (Hayward, CA, USA). All assays were preformed according to the manufacturers’ instructions. The plasma concentrations of TNF-α and IFN-γ were examined using a Mouse TNF-alpha Colorimetric ELISA Kit (Thermo, Fisher Scientific, Waltham, MA, USA) and a Mouse IFN-gamma Colorimetric ELISA Kit (Thermo, Fisher Scientific), respectively, according to the manufacturers’ instructions.

### Cytokine gene expression analysis in dsRNAs-exposed splenocytes

Splenic immune cells (splenocytes) were prepared from intact ICR mice (male; 10-week-old) and subjected to analysis of cytokine gene expression. Briefly, spleens isolated from ICR mice were mashed with a syringe plug and passed through a 70-µm nylon cell strainer (BD Bioscience) for elimination of connective tissues and cell debris. These cells were then suspended in PBS. Approximately 3 ml of the cell suspension was layered onto an equal volume of HistoPaque-1083 (Sigma-Aldrich) and subjected to centrifugation at 400 × *g* for 30 min at room temperature. After centrifugation, a visible interlayer containing splenocytes was collected and washed with RPMI-1640 medium. The collected cells were seeded onto 24-well culture plates at a cell density of 5 × 10^5^ cells/well in RPMI-1640 containing 10% FBS and exposed to a defined concentration of poly(I:C) (Amersham Pharmacia Biotech, Uppsala, Sweden) and siRNAs [0, 1, 10, or 100 nM (final concentration)]. After a 24-h exposure (incubation), total RNAs were extracted from the splenocytes using TRIzol reagent (Invitrogen), according to the manufacturer’s instructions; RNA samples were used as a template for cDNA synthesis, as described above. The cDNAs were examined by real-time PCR (qPCR) using an AB 7300 Real Time PCR System (Applied Biosystems) and a TaqMan Universal PCR Master Mix, together with Assays-on-Demand Gene Expression products, according to the manufacturer’s instructions (Applied Biosystems). The Assays-on-Demand Gene Expression products used and their assay IDs were as follows: *Tumor necrosis factor-alpha* (*Tnf-α*), Mm00443258_m1; *Interferon-alpha* 2 (*Ifn-alpha2*), Mm00833961_s1; *Ifn-gamma*, Mm01168134_m1; and *Gapdh*, Mm99999915_g1*.*

### Cytotoxicity assay of dsRNAs-exposed splenocytes against naïve PC-3 cells

Splenocytes were prepared from intact ICR mice as described above, seeded onto 96-well culture plates at a cell density of 50, 25, 12.5, or 6.25 × 10^5^ cells/well, and exposed to 100 nM of poly(I:C) and siRNAs (final concentration). After a 24-h exposure (incubation), naïve PC-3 cells (≈1 × 10^5^ cells/well) were added to each well, and the splenocytes and PC-3 cells were co-cultured for 6 h as effector and target cells, respectively. Lactate dehydrogenase (LDH) released from PC-3 cells into culture media was examined using a CytoTox 96 Non-Radioactive Cytotoxicity Assay (Promega), according to the manufacturer’s instructions.

### Cytotoxicity assay of splenocytes prepared from siRNA-treated cancer mouse models against naïve PC-3 cells

Splenocytes were prepared from mice with xenografts that had been treated with siRNAs; these splenocytes were seeded onto 96-well culture plates at a cell density of 50, 25, 12.5, or 6.25 × 10^5^ cells/well as described above. To each well, naïve PC-3 cells (≈1 × 10^5^ cells/well) were immediately added, and the splenocytes and PC-3 cells were co-cultured for 6 h. After the co-culture, the LDH released from PC-3 cells was examined as described above.

### IC50 analysis of EGFR-tyrosine kinase inhibitors (EGFR-TKIs)

Gefitinib (JS Research Chemicals Trading e. Kfm., Schleswig Holstein, Germany) and erlotinib (Cayman Chemical Company, Ann Arbor, MI, USA) were used as EGFR-TKIs and dissolved in dimethyl sulfoxide (DMSO) (Sigma-Aldrich). Cultured cells were exposed to increasing amount of each EGFR-TKI, but the concentration of DMSO as solvent remained unchanged (0.02%). After a 3-day exposure, cell viability was examined using a CellTiter 96 *AQ*ueous One Solution Cell Proliferation Assay (Promega), according to the manufacturer’s instructions.

### Oral administration of gefitinib

Subcutaneous tumor model mice that were established with PC-3/luc cells, were treated by gavage administration of gefitinib at a dose of 0, 50, or 100 mg/kg b.w [21,22]. . The gavage administration was performed once a day on weekdays, and the treatment was carried out for three weeks. Tumor growth was monitored by an IVIS imaging system once a week.

### Statistical analysis

One-way analysis of variance (ANOVA) followed by the Dunnett’s test was performed in the following assessments: IC50 assay (dose-dependent cytotoxicity assay), splenocytes-mediated cytotoxicity assay, hematological assessments, cell viability assay, and gene expression analyses (*Egfr, Ifn-α, Ifn-γ*, and *Tnf-α*).

Wet weight of tissues, blood cell counts, and hematocrit values were analyzed by one-way ANOVA, and body weight was analyzed by two-way ANOVA. One-way ANOVA followed by Tukey-Kramer test was performed to assess the effects of siRNAs on tumor suppression and the differences in the CD31- and Ki67-positive cells. The differences in the wet weight of lung samples and in the luminescent signal intensities of xenografts were analyzed by Student’s *t*-test (two-tailed). For all statistical analyses, the α-value was set at 0.05.

## Results

### Oncogenic EGFR allele-specific RNAi and inhibition of cancer cells

We designed siRNAs that targeted the disease-causing *EGFR* deletions for ASP-RNAi (Table S1). An *in vitro* assay system was used to select siRNAs that conferred a strong allele-specific silencing of disease-causing *EGFR* alleles [9–13]. This assay depends upon two reporter alleles of the *Photinus* and *Renilla* luciferase genes; these alleles encode mutant and normal *EGFR* sequences in their 3’-untranslated regions (Table S2). The effects of test siRNAs on target mutant alleles and also on non-target normal alleles were simultaneously examined. Based on *in vitro* findings (Figure S1), we selected two competent siRNAs, si747/49_3D8 and si746/50_3D4, that specifically targeted the *L747_E749del, A750P* and *E746_A750del* mutations, respectively. Each siRNA discriminated between the oncogenic and normal *EGFR* alleles, and induced a potent inhibition of the oncogenic allele (Figure 1A, B). Introduction of the respective siRNA into PC-3 (see **Materials and Methods**) or PC-9 human lung adenocarcinoma cells, which carried *L747_E749del, A750P* and *E746_A750del*, respectively, resulted in a strong inhibition of cell proliferation, induction of cell death, or both (Figure 1C). Dose-dependent effects of the siRNAs on cell viability indicated that si747/49_3D8-treated PC-3 cells exhibited survival curves similar to those of si746/50_3D4-treated PC-9 cells (si747/49_3D8, IC50 = 34 nM; si746/50_3D4, IC50 = 27 nM) (Figure 1D): this suggests that these two allele-specific siRNAs have similar cytosuppressive effects on the respective cell types which differ from each other in the sensitivity to EGFR-TKIs (Figure S2). Similar results were also obtained when siEGFR targeting both the mutant and wild-type *EGFR* alleles was used instead of the allele-specific siRNAs (Figure S3). Therefore, the findings suggested that RNAi knockdown of oncogenic *EGFR* alleles probably allowed for inhibition of cancer cells possessing the oncogenic alleles, regardless of the sensitivity of the cells to EGFR-TKIs.

**Figure 1:** Oncogenic allele-specific RNAi. (**A**) Specific inhibition of mutant *EGFR* reporter alleles by ASP-RNAi. The effects of allele-specific siRNAs, si747/49_3D8 and si746/50_3D4, on expression of the target *L747_E749del, A750P* and *E746_A750del EGFR* mutant reporter alleles, respectively, and of the normal reporter alleles were examined using IC50 analysis (details in Methods). The IC50 values of the siRNAs for inhibition of the mutant and wild-type alleles are indicated (n=4, mean ± SDs). (**B**) Specific suppression of endogenous or oncogenic *EGFR* alleles. The si747/49_3D8 and si746/50_3D4 siRNAs were introduced into PC-3 and PC-9 human adenocarcinoma cells possessing the *L747_E749del, A750P* or *E746_A750del* mutations, respectively; endogenous *EGFR* mRNAs were examined using RT-PCR. Cells transfected with siControl (non-silencing siRNA) were studied as a control. M: DNA marker. (**C**) ASP-RNAi-mediated inhibition of PC-3 and PC-9 cell proliferation. Single siRNAs were transfected into PC-3 and PC-9 cells; subsequently, the cells were stained with Hoechst 33342 (blue) and propidium iodide (PI) (red) at the indicated time points, and examined using a fluorescent microscope. The numbers of total and dead cells were counted in four different 1-mm^2^ areas. The data are averages of the four counts (± SDs; *P < 0.05). (**D**) Effect of allele-specific siRNAs on cell viability. Viability of PC-3 and PC-9 cells following treatment with the indicated siRNA was examined using the MTS assay (n=4, mean ± SDs).

Western blot analyses of protein components of the EGFR signal pathway furthermore revealed that the phosphorylation level of EGFR, AKT, and ERK1/2 was markedly reduced in PC-3 and PC-9 cells subjected to the specific inhibition of oncogenic *EGFR* alleles by ASP-RNAi (Figure S4). Another intriguing point in the expression profile is that there was no marked difference in the signal intensity of whole EGFR between oncogenic allele-specific siRNAs and siControl although the specific inhibition of the target oncogenic alleles appeared to occur. This might be caused by a predominant expression of normal EGFR or by a compensational expression of normal *EGFR* during a specific suppression of mutant *EGFR*.

### ASP-RNAi Treatment of Subcutaneous Tumors

We examined the *in vivo* effects of ASP-RNAi treatment with the si747/49_3D8 siRNA and two distinct models of cancerous tumors (subcutaneous tumors and lung tumors) in mice. Both types of tumors were established by subcutaneous inoculation and tail vein injection of PC-3 cells or PC-3/luc cells that carried a marker gene, *firefly luciferase*, into athymic nude mice. We also tried to establish subcutaneous and lung tumor models using PC-9 cells, but without success.

The subcutaneous tumors were subjected to a one-time intratumoral administration of si747/49_3D8 siRNA. Tumor growth was clearly suppressed by si747/49_3D8 administration in a dose of more than 1.0 mg/kg b.w, but not in a dose of less than or equal to 0.5 mg/kg b.w (Figure 2 and Figure S5, S6). In suppressed tumors, the expression of the mutant *EGFR* (Figure S7) and the phosphorylation level of EGFR, AKT, and ERK1/2 (Figure 2E) were markedly reduced, consistently indicating the inhibition of the EGFR signal pathway *in vivo*. In addition, si747/49_3D8-treated (ASP-RNAi-treated) mice had much fewer Ki67-positive or CD31-positive cells than did siControl- (non-silencing siRNA) or non-siRNA-treated mice (Figure S5C). Ki-67 and CD31 are markers of proliferation and vascular endothelial tissue, respectively. Therefore, these findings indicated that tumor growth and angiogenesis were markedly inhibited in the ASP-RNAi-treated mice.

**Figure 2:** Effects of ASP-RNAi on tumor growth. (**A**) Schematic drawing of the experimental plan. s.c.: subcutaneous. (**B**) *In vivo* luminescent imaging. Subcutaneous tumor models were established with PC-3/luc cells and siRNAs at indicated doses were administered according to the experimental plan (A). Tumors were monitored by an IVIS imaging system. (**C**) Tumor growth. Luminescent intensities of the tumors treated with siRNAs were quantified and analyzed (mean ± SDs, n = 5 mice/group). (**D**) Wet weight of tumors treated with siRNAs. Three weeks after treatment (Day 28), the treated tumors were isolated and their wet weight was measured [mean ± SDs; n = 5 mice/group; *P < 0.05 by Dunnett’s test (vs. siControl)]. (**E**) Western blot analysis. Subcutaneous tumors were treated with 2.0 mg/kg b.w. of si747/49_3D8 (red box) or siControl (open box). Three days after treatment (Day 10), the treated tumors were isolated and examined by Western blotting using indicated antibodies. (**F**) Plasma biochemical parameters in mice treated with siRNAs. Plasma specimens were prepared from treated mice at Day 28, and subjected to plasma biochemical analyses to examine alkaline phosphatase (ALP), total protein (TP), GPT, GOT, and total (T-), direct (D-) and indirect (I-) bilirubin (BIL). Significant difference in each parameter was examined by Dunnett’s test as in D. n.s., no significant difference. (**G**) Body weight. Body weight of the treated mice was measured at Day 28. Statistical analysis was carried out as in F.

To assess the effects of siRNA treatment on immune responses and physiological homeostasis, several indicators—including body weight, hematological parameters, plasma cytokines, and immune responses of isolated splenocytes—were monitored (Figure 2F, G, Figure S8, S9 and Table S3, S4). Based on the data, there were no significant differences between si747/49_3D8-treated and siControl- or non-siRNA-treated mice with regard to any indicator, suggesting that none of the detrimental immune responses and biological adverse effects, which were associated with siRNA administration, were activated in these mice.

### ASP-RNAi treatment of lung cancer models

Cancerous tumors established by tail vein injection of PC-3/luc cells were successfully engrafted in the lung, i.e., they looked like lung cancer tumors (Figure 3A). Mice with established lung tumors were subjected to two rounds of systemic administration of si747/49_3D8 or siControl, and the luciferase activity (luminescence) of the engrafted tumor cells was monitored via *in vivo* imaging. The amount of luminescence in the si747/49_3D8-treated mice was significantly lower than that in the mice treated with siControl (Figure 3A and Figure S10).

**Figure 3:** Effects of systemic siRNA administration on tumor growth in lung cancer models. (**A**) *In vivo* luminescent imaging. PC-3/luc cells were intravenously administered to nude mice and examined using an IVIS imaging system 5 days after cell injection. PC-3/luc-positive mice were randomly divided into two groups, and subjected to systemic administration of indicated siRNAs twice (Day 5 and 7) via the lateral tail vein. The treated mice were examined using the IVIS imaging system; photographic images of luminescent signals at Day 5 and 10 (after cell injection) are shown (left panels). Box plots represent the luminescent intensities of the treated mice at Day 5 and 10 (right panels) [n = 5 mice/group; *P < 0.05 by Student’s *t*-test (two-tailed); n.s., no significant difference]. (**B**) Lung tissues isolated from siRNA-treated mice. Lung tissues were isolated from PC-3-bearing mice treated with the indicated siRNAs, and the wet weights were measured [mean ± SDs; n=5 mice/group; *P < 0.05 by Student’s *t*-test (two-tailed)]. (**C**) Histological analysis of lung tissues. Cryosections of lung tissue were prepared from PC3-bearing mice treated with the indicated siRNAs; cryosections were stained with conventional hematoxylin and eosin solution. (**D**) *In vivo* imaging of active caspase. Six hours after administration of the indicated siRNAs on Day 5, VivoGlo Caspase 3/7 substrate (Promega) was administrated intraperitoneally to the treated mice; *in vivo* imaging and subsequent imaging analysis were carried out. Box plots represent luminescent intensities [n = 6 mice/group; *P < 0.05 by Student’s *t*-test (two-tailed)].

Wet-weight measurements indicated that lungs of siControl-treated mice were significantly heavier than those of si747/49_3D8-treated mice (Figure 3B). Based on histological analysis, tumors had clearly formed in the lung parenchyma of the siControl-treated mice, but fewer tumors had formed in the lungs of si747/49_3D8-treated mice (Figure 3C). Accordingly, the greater wet-weight of the lungs from siControl-treated mice, relative to those from si747/49_3D8-treated mice, may have been due to unsuppressed tumor growth in the siControl-treated mice.

An *in vivo* caspase assay further revealed that caspase activity was elevated in the si747/49_3D8-treated mice (Figure 3D); this indicates that caspase activity and subsequent apoptosis may have been involved in tumor suppression in si747/49_3D8-treated mice. Therefore, the findings of ASP-RNAi treatment for the lung and subcutaneous tumors strongly suggested that the si747/49_3D8 siRNA and the consequent ASP-RNAi effectively suppressed tumor growth *in vivo*.

### Adverse effects of suppression of normal *Egfr* in normal mice

To verify that si747/49_3D8 had no adverse effects on normal cells or tissues *in vivo* and to verify that RNAi-mediated suppression of the normal *EGFR* gene did have such adverse effects, we administered si747/49_3D8, siControl, or siEgfr, which targets normal mouse *Egfr* (Figure S11, S12), to normal ICR mice. After three systemic administrations of the individual siRNAs, the treated ICR mice were examined. Plasma alkaline phosphatase levels were significantly elevated in siEgfr-treated mice than in any other group of mice, and a trend toward increasing in the level of total- and indirect-bilirubin was also observed in the siEgfr-treated mice (Figure 4A); these findings may suggest damage to the liver, biliary tract dysfunction, or both.

**Figure 4:** Adverse effects of knockdown of normal *Egfr* in normal ICR mice. (**A**) Plasma analyses. siEgfr siRNA targeting the wild-type mouse *Egfr* gene, another siRNA (as indicated), or delivery vehicle was administered 3 times, on Days 1, 3, and 5, to 10-week-old ICR mice via the lateral tail vein. The day after administration, measurement of body weight was carried out (Table S5). Two days after the last administration, the mice were subjected to hematological analyses (Table S6) followed by separation of blood plasma. The plasma specimens were examined as in Figure 2. Examined biochemical parameters are indicated (n=4 mice/group; mean ± SDs; * *P*<0.05 by Tukey-Kramer test; n.s., no statistical significance). (**B**) TUNEL assay. Cryosections of intestinal tissue were prepared from ICR mice that had been treated with the indicated siRNAs; cryosections were examined using a TUNEL assay. A marked increase in intestinal apoptosis was detected in the siEgfr-treated ICR mice.

Most interestingly, TUNEL assays revealed that apoptosis was significantly more frequent in intestines of siEgfr-treated mice than in those of any other group of mice (Figure 4B); therefore, *EGFR* may have a vital role in normal intestinal cells and tissue. As for si747/49_3D8-treated mice, they did not differ significantly from mice treated with either vehicle or siControl in any of the assays performed (Figure 4, Figure S13, S14 and Table S5, S6); the findings were consistent with those obtained from subcutaneous tumor model mice treated with si747/49_3D8 (Figure 2, Figure S8, S9 and Table S3, S4).

Similar results were also obtained when subcutaneous tumor model mice were treated with gefitinib (Figure 5). Gefitinib treatment worked for the suppression of tumor growth, whereas intestinal apoptosis was significantly frequent in the mice treated with a high dose of gefitinib (100 mg/kg b.w.), and also the treated mice exhibited an increasing trend in the level of plasma alkaline phosphatase, GOT, GPT and (total-, direct- and indirect-) bilirubin. Moreover, it is noteworthy that gefitinib-treated mice developed significant weight loss. As for other side effects such as additional sebostatic skin reactions, paronychia and changes in the hair structure, which may occur in patients treated by TKIs, such a symptom was not observed in either gefitinib or siRNA treated mice by our visual inspection in this study.

**Figure 5:** Effects of gefitinib on tumor growth. (**A**) Schematic drawing of the experimental plan. p.o.: per os (oral administration). (**B**) *In vivo* luminescent imaging. Subcutaneous tumor models were established with PC-3/luc cells as in Figure 2, and gefitinib was administered at the indicated doses. Photographic images of luminescent signals at Day 7 and 28 after the inoculation of PC-3/luc cells are shown. (**C**) Tumor growth. Luminescent intensities of the tumors treated with gefitinib were quantified and analyzed (n = 5 tumor models/group). Error bars represent SDs. (**D**) Wet weight of the tumors treated with gefitinib. Three weeks after treatment (Day 28), the treated tumors were isolated and wet weight was measured. A significant difference against the vehicle control group (open bar) is indicated by an asterisk [*P < 0.05 by Student’s *t*-test (two-tailed)]. Error bars represent SDs. (**E**) Examination of plasma biochemical parameters in the treated mice. Plasma specimens were prepared from the mice at Day 28, and subjected to plasma biochemical analyses as in Figures 2 and 4 [n = 5 mice/group; mean ± SDs; *P* < 0.05 by Dunnett’s test (vs. siControl); n.s., no significant difference]. (**F**) Body weight. Body weight of the treated mice was measured at Day28 [n = 5 mice/group; mean ± SDs; *P < 0.05 by Dunnett’s test (vs. siControl)]. (**G**) TUNEL assay. Cryosections of intestinal tissues were prepared from model mice treated with gefitinib (0, 50, 100 mg/kg b.w.) at Day 28 as in Figure 4, and the cryosections were examined by a TUNEL assay.

When taken together, the findings presented here indicated that the suppression or functional inhibition of normal EGFR had adverse effects on normal tissues and organs, and that si747/49_3D8, which is specific for an oncogenic *EGFR* allele, caused no harm to normal tissues or organs composed of cells with no target RNA for si747/49_3D8. 

## Discussion

Specific inhibition of oncogenic alleles may be a promising approach that will lead to safe cancer therapies, although the strategy may be confined to cancer cases having causative oncogenic mutations. Our current study demonstrated that ASP-RNAi allowed for specific inhibition of oncogenic *EGFR* alleles carrying disease-causing mutations without affecting the normal *EGFR* allele (Figure 1), and provided a highly effective antitumor activity, both *in vivo* and *in vitro* (Figures 1-3). The inhibition of oncogenic EGFR signaling such that the phosphorylation level of EGFR, AKT, and ERK1/2 is markedly reduced by specific silencing of oncogenic EGFR, may trigger cell death involving a caspase activation [23,24] (Figures 2E, 3D and Figure S4), thereby suppressing tumor cell growth. Therefore, our findings suggest that specific inhibition of oncogenic *EGFR* alleles may be a promising strategy for treatment of various cancers involving causative oncogenic mutations.

ASP-RNAi treatment allows for suppression of cancer cells regardless of the sensitivity of the cells to EGFR-TKIs (Figure 1D and Figure S2); this is because RNAi silencing is mechanistically different from EGFR-TKI-mediated inhibition, and the feature of ASP-RNAi may permit an anticancer therapy for patients with cancers resistant to EGFR-TKIs. Therefore, it is possible that ASP-RNAi and EGFR-TKIs treatments may help each other in anticancer therapies.

A major benefit of ASP-RNAi treatment is that it targets a specific disease-causing allele and is therefore harmless to any cell lacking that allele, e.g., normal cells. Our current findings consistently proved that ASP-RNAi treatment caused no harm to normal cells or tissues (Figure 4, Figure S13, S14 and Tables S3-S6). In addition, we further revealed evidence that either the suppression of normal EGFR by a conventional RNAi or a functional inhibition of the EGFR-tyrosine kinase activity by gefitinib had adverse effects *in vivo*; particularly, intestinal apoptosis was noticeable in both the RNAi- and gefitinib-treated mice (Figures 4, 5). When taken together, our current findings suggest that specific inhibition of oncogenic *EGFR* alleles without affecting the normal *EGFR* allele is a key element for a safe anticancer treatment, and that ASP-RNAi may be capable of becoming such a safe and effective anticancer therapeutic method.

ASP-RNAi treatment is a personalized medicine, and approximately a half of NSCLC cases carrying *EGFR* mutations, regardless of the sensitivity to EGFR-TKIs, may be treatable with the current ASP-RNAi method. Diagnosis including an *EGFR* mutation typing is absolutely necessary for providing an appropriate ASP-RNAi treatment. Therefore, the advancement of an early diagnostic technology as well as a drug delivery system of siRNAs is vital to the realization of ASP-RNAi treatment; and extensive studies on these issues need to be carried out in the future. 

## Supporting Information

Figure S1 **Assessment of siRNAs against EGFR mutant alleles.** SiRNAs against the *L747_E749del*, *A750P*, and *E746_A750del EGFR* mutant alleles were designed and chemically synthesized; the sequences of the designed siRNAs are shown in Table S1. The effects of the siRNAs on specific silencing against the EGFR mutant reporter alleles and off-target silencing against the normal reporter allele were simultaneously examined by our in vitro assessment system. The ratios of the mutant and normal reporter activities in the presence of test siRNAs were normalized to the control ratio obtained with non-silencing siRNA (siControl) as 1. Similar results were also obtained when the luciferase reporter genes were exchanged between the normal and mutant reporter alleles (A vs. B; C vs. D). Data are averages of four independent determinations. Error bars represent SDs.
(TIF)

Figure S2 **Effects of gefitinib and erlotinib, EGFR-tyrosine kinase inhibitors, on cell viability.** Cell viability of PC-3 and PC-9 cells after treatment of gefitinib or erlotinib was examined by means of a MTS assay as in Figure 1D. The results indicated that PC-9 cells were sensitive to each inhibitor (gefitinib, IC50 = 79 nM; erlotinib, IC50 = 82 nM), whereas PC-3 cells were less sensitive to the inhibitor (gefitinib, IC50 = 3.8 µM; erlotinib, IC50 = 1.3 µM). Data are averages of four independent measurements. Error bars represent SDs.
(TIF)

Figure S3 **Effects of *EGFR* knockdown on cell viability.** (**A**) *EGFR* knockdown in PC-3 and PC-9 cells. The Silencer^®^ Select Validated siRNA (Applied Biosystems) against normal human *EGFR* gene (siEGFR) was purchased and transfected into PC-3 and PC-9 cells. The cells were stained with Hoechst 33342 (blue) and propidium iodide (PI) (red), and the cells positive for each dye were counted in four different 1-mm^2^ areas as in Figure 1C. The data are averages of the four counts. (**B**) Cell viability. Viability of PC-3 and PC-9 cells following treatment with the indicated siRNAs was examined using a MTS assay as in Figure 1D. Data are averages of four independent measurements. Error bars represent SDs.
(TIF)

Figure S4 **Western blot analysis.** PC-3 and PC-9 cells were subjected to transfection with indicated siRNAs. Two days after transfection, cell extracts were prepared and examined by Western blotting using the indicated antibodies. The results indicated that the level of phosphorylated EGFR (pEGFR), AKT (pAKT), or ERK1/2 (pERK1/2) was markedly reduced in the cells treated with si747/49_3D8 or si746/50_3D4. In addition, a marked reduction of the oncogenic EGFR deletion mutant under ASP-RNAi was confirmed by an E746_A750del EGFR specific antibody in PC-9 cells.
(TIF)

Figure S5 **Effects of intratumoral siRNA administration on tumor growth.** (**A**) Tumor growth after siRNA administration. Engrafted tumors were subjected to a one-time intratumoral siRNA administration (1.0 mg/kg b.w.) as in Figure 2 and measured with a caliper. Five different tumors in five different individuals from each treatment group were examined. Error bars represent SDs. (**B**) Wet weight of isolated tumors. Three weeks after siRNA administration, tissues were isolated and measured by wet weight. Error bars represent SDs. Significant differences between the si747/49_3D8-treated group (tumors) and any of the other groups are indicated with an asterisk (*P* < 0.05). (**C**) Immunohistochemical analysis. Cryosections of tumors were prepared from each group (indicated) subjected to staining with anti-Ki67 IgG (red), anti-CD31 IgG (green), and Hoechst 33342 (blue), and examined using a fluorescent microscope (left panels). The Ki67- or CD31-positive area was calculated and normalized to a Hoechst-stained area in the same region, and four different cryosections from each group were examined. The data were further normalized to the data of the non-treated group, which was set as 100%. Error bars represent SDs. Significant differences between the si747/49_3D8-treated group and any of the other groups are indicated with an asterisk (*P* < 0.05).
(TIF)

Figure S6 **siRNA treatment in mouse xenograft models.** Xenograft models established with PC-3/luc cells were treated by siRNAs at the indicated doses. Tumor growth was monitored by an IVIS imaging system (Xenogen) and analyzed using a Living Imaging software (Xenogen) as in Figure 2.
(TIF)

Figure S7 **Specific suppression of mutant *EGFR* in xenograft tumors.** Subcutaneous xenograft tumors were subjected to intratumoral injection of si747/49_3D8 or siControl (1.0 mg/kg b.w.). Three days after treatment (upper right panel), total RNAs were extracted from treated tumors, and examined by RT- semi-quantitative PCR for both normal and mutant *EGFR* transcripts, followed by polyacrylamide gel electrophoresis and ethidium bromide staining. Xenograft tumors before treatment (upper left panel) were also examined by the same method. The results obtained from three independent tumors (experiments) were indicated (upper panel). To further analyze the expression level of normal and mutant *EGFR*, PCR bands were examined by a densitometer. Relative expression ratios were calculated and indicated in a lower panel. Error bars represent SDs. n.s., no statistical significance. * *P* < 0.05 by Student’s *t*-test (two-tailed).
(TIF)

Figure S8 **Immunostimulatory potential of RNA duplexes.** (**A**) Schematic drawing of the experiment design. Splenocytes were prepared from intact ICR mice and exposed to double-stranded RNAs (dsRNAs). After a 24h-exposure, gene expression assay was carried out. (**B**) Cytokine gene expression in splenocytes treated with dsRNAs. Splenocytes were exposed to siControl, si746/50_3D4, si746/49_3D8, and poly(I:C) (as a positive control) at final concentrations of 0, 1, 10, and 100 nM. After a 24h-exposure, total RNA was extracted. The expression levels of *interferon-α* (*Ifn-α*), *Ifn-γ*, and *tumor necrosis factor-α* (*Tnf-α*) were examined by RT-qPCR followed by delta Ct analysis with the Ct of *Gapdh* as an internal control. The data were further normalized to the data obtained from naïve splenocytes (0 nM dsRNA) as 1 (indicated by dotted lines in graphs). Data are averages of four independent examinations (± SDs; * *P* < 0.05 by ANOVA followed by Dunnett’s test). (**C**) Schematic drawing of the experiment design. Splenocytes (Effector) were exposed to dsRNAs for 24 h, and PC-3 cells (Target) were added to the treated splenocytes. After a 6h-coculture, a LDH assay was carried out. (**D**) Cytotoxicity of dsRNAs-exposed splenocytes against intact PC-3 cells. LDH released from PC-3 (target) cells that were lysed by cytotoxic splenocytes (effector) was investigated. E/T ratios [splenocytes (effector) /PC-3 cells (target)] are indicated. Data are averages of four independent examinations. Error bars represent SDs. The data obtained at 50 E/T ratio were statistically analyzed against the data with non-treatment by ANOVA followed by Dunnett’s test (* *P* < 0.05). Note that no significant difference was detected between the non-treatment splenocytes and any of the siRNA-exposed splenocytes.
(TIF)

Figure S9 **Plasma cytokine level and cytotoxicity of splenocytes in siRNAs-treated mice.** (**A**) Plasma cytokine level. Xenograft mouse models were subjected to administration of the indicated siRNAs or delivery vehicle as in Figure S5. Three weeks after administration, the level of TNF-α and IFN-γ in plasma prepared from the treated xenograft models were examined by using an ELISA. Data are averages of five individual data in each treated group. Error bars represent SDs. n.s., no statistical significance. (**B**) Cytotoxicity of splenocytes prepared from siRNAs-treated mice. The experiment design is schematically indicated in an upper panel. Splenocytes prepared from the treated xenograft models (indicated) were subjected to a cell-mediated cytotoxicity assay as in Figure S8D. Data are averages of four independent examinations. Error bars represent SDs. The data presented here are consistent with the results of Figure S8, and both the results strongly suggest that si747/49_3D8 has no immunostimulating activity.
(TIF)

Figure S10 **Effects of competent siRNA on tumor suppression in lung cancer models.** Two independent *in vivo* experiments (**A**, **C**) described in Figure 3 were carried out. All the experimental techniques and conditions were the same as Figure 3. The data of Figure 3 were derived from the first experimental data (**A**). Line graphs (**B** and **D**) represent the luminescent intensities of the mice (A and C, respectively) examined at the indicated time points (Day) relative to the day of administration of PC-3/luc cells into mice (Day 0). Data are averages of 5 or 6 individual mice data in each group (± SEMs).
(TIF)

Figure S11 **RNAi knockdown of the endogenous normal *Egfr* gene.** Silencer^®^ Select Validated siRNAs (Applied Biosystems) against normal mouse *Egfr* gene (siEgfr#01 and #02) were used and transfected to mouse Neruo2A (N2a) cells. 24 h after transfection, the expression level of endogenous normal *Egfr* was examined by RT-qPCR and analyzed as in Figure S8B. The normalized expression levels were further normalized to the data obtained in naïve N2a cells (Non-treatment) as 1. Data are averages of four independent determinations (± SDs; * *P* < 0.05 by ANOVA followed by Dunnett’s test). The results indicate that either siEgfr#01 or #02 can confer a strong inhibition against endogenous normal mouse *Egfr*, whereas si747/49_3D8 as well as siControl induces little or no suppression against the mouse *Egfr* gene. The siEgfr#01 referred to as “siEgfr” was further used in subsequent studies (Figure 4 and Figures S12-S14).
(TIF)

Figure S12 **Immunostimulatory potential of siEgfr.** The same experiments as in Figure S8 were carried out using siEgfr. The experimental plans (**A**, **C**), techniques and conditions (**B**, **D**) other than using siEgfr were the same as Figure S8. (**B**) Cytokine gene expression in splenocytes treated with dsRNAs. Examined genes are indicated. Data are averages of four independent examinations (± SDs; * *P* < 0.05 by ANOVA followed by Dunnett’s test). (**D**) Cytotoxicity of dsRNAs-exposed splenocytes against intact PC-3 cells. The data obtained at 50E/T ratio were statistically analyzed against the data of non-treatment by ANOVA followed by Dunnett’s test (* *P* < 0.05). The results suggested that siEgfr triggered no immune stimulation.
(TIF)

Figure S13 **Plasma cytokine level and cytotoxicity of splenocytes in siRNAs-treated ICR mice.** The experiments similar to Figure S9 were performed using siEgfr and ICR mice. (**A**) Plasma cytokine level. The indicated siRNAs or delivery vehicle were administered 3 times every second day to 10-week-old ICR mice as in Figure 4. Two days after the last administration, plasma and splenocytes were prepared from the treated ICR mice. The level of TNF-α and IFN-γ in plasma was examined by an ELISA and analyzed as in Figure S9. Error bars represent SDs. n.s., no statistical significance. (**B**) Cytotoxicity of splenocytes prepared from siRNAs-treated ICR mice. Splenocytes prepared from the treated ICR mice (indicated) were subjected to a cytotoxic assay as in Figure S9. Data are averages of four independent examinations. Error bars represent SDs. The presented data were consistent with the results of Figure S12, and both the results indicated that siEgfr had no immunostimulating activity.
(TIF)

Figure S14 **Histological examination of tissues from siRNAs-administered ICR mice.** The indicated tissues derived from the same ICR mice used in Figure 4 were further subjected to histological examination using an H&E staining. As a result, histological alteration was hardly detected among the specimens in each examined tissue.
(TIF)

Table S1 **The sequences of synthetic siRNAs against *EGFR* deletions.**
(PDF)

Table S2 **Synthetic DNA oligonucleotides used in the construction of reporter alleles.**
(PDF)

Table S3 **Hematological parameters in xenograft mouse models treated with siRNAs at Day 28.** The same mice investigated in Figure S5 were examined at Day 28. Data are averages of 5 individual specimens in each group (±SD). No significant difference was observed by one-way ANOVA.
(PDF)

Table S4 **Hematological parameters in xenograft mouse models treated with siRNAs.** Examined mice were the same as the mice investigated in Figure 2. Data are averages of 5 individual specimens in each group (±SD). No significant difference was observed by one-way ANOVA.
(PDF)

Table S5 **Body weight of ICR mice treated with siRNAs.** The agents indicated were intravenously injected three times every second day to ICR mice. Data are averages of 5 individual mice per group (±SD). No significant difference was observed by two-way ANOVA.
(PDF)

Table S6 **Hematological parameters in ICR mice treated with siRNAs.** The same mice investigated in Figure 4 and Table S5 were examined at Day 6. Data are averages of 5 individual specimens in each group (±SD). No significant difference was observed by one-way ANOVA.
(PDF)
